# WeChat-Based Comprehensive Education on Egg White Protein Intake for Patients Undergoing Peritoneal Dialysis: A Combined Prospective and Retrospective Study

**DOI:** 10.1155/2022/5651992

**Published:** 2022-07-31

**Authors:** Tianzhao Han, Yunlei Deng, Dayong Quan, Dan Wu, Shuxin Xiao, Rong Gong

**Affiliations:** Department of Nephrology, Third People's Hospital of Chengdu, The Second Chengdu Affiliated College of Chongqing Medical University, Sichuan 610031, China

## Abstract

Protein malnutrition is a well-described complication of peritoneal dialysis (PD), a standard mode of treatment for end-stage renal disease (ESRD), and contributes to morbidity, treatment failure, and mortality. To assess the usefulness of WeChat-based education for ensuring optimal protein intake through the consumption of egg white protein, 140 young and middle-aged patients undergoing PD are assigned to either the intervention group or the control group. The results show that reinforcing comprehensive PD education using WeChat can improve nutritional parameters, clinical parameters, and quality of life.

## 1. Introduction

Peritoneal dialysis (PD) is a common renal replacement therapy (RRT). Several young and middle-aged patients with end-stage renal disease (ESRD) chooses PD as the first choice of RRT in China, as it is simple and be performed at home. However, because of the loss of albumin and absorption of glucose from the dialysate, PD patients always have a poor appetite. Along with the effect of uremic toxins, poor appetite reduces the protein-energy intake, which is strongly associated with malnutrition, low serum albumin, and microinflammation [1, 2]. Protein energy wasting (PEW) is a common and severe complication in PD patients. Furthermore, the presence of hypoalbuminemia has been shown to predict all-cause mortality and peritonitis risk in PD patients [3, 4]. The International Society of Renal Nutrition and Metabolism (ISRNM) recommends sufficient dietary protein intake (DPI) for PD patients. At least 50% of the dietary protein should be of high biological value [5]. Protein-rich foods are a major source of dietary phosphorus. Excess DPI results in hyperphosphatemia related to adverse clinical outcomes, and its reduction may lead to malnutrition and inflammation, which result in increased morbidity and mortality in patients on maintenance dialysis [6, 7]. Consequently, foods with low phosphorus-to-protein ratios may balance the intake of protein and phosphate. Clinicians face a considerable challenge in helping PD patients to achieve adequate protein intake with restricting dietary phosphorus. Educational interventions play a key role in helping individuals manage their “renal” diets and become active participants in therapy [8]. However, in conventional education, performed through telephone or oral outpatient follow-up, it is difficult to achieve the expected dietary intake and treatment outcomes for PD patients. Furthermore, as young and middle-aged individuals undertake family responsibility, it is important to improve their quality of life.

In China, WeChat, a comprehensive, large-scale, instant, and free network social media platform, is widely used among young individuals, including those receiving PD for life-sustaining RRT. WeChat can be used to send a vast amount of data through text messages, image sharing, voice communication, and video consultation. Several clinical studies have used WeChat as a tool for conducting educational health interventions [9, 10]. Herein, we used WeChat to provide intensive education to young PD patients to improve their nutritional status and treatment outcomes for long-term management of PD. We design an education module that includes conventional education and innovative comprehensive PD education, with emphasis on egg white-based optimal protein intake, which has the lowest phosphorus-to-protein ratio [11, 12].

The rest of this paper is organized as follows: Section 2 discusses related research and summary analysis, followed by the methods of clinical diagnosis and data statistics in Section 3. The comparative analysis and data statistics are in Section 4.  Section 5 concludes the paper with future research and summary.

## 2. Related Work

Health education for patients with ESRD treated with PD is an integral component of management that contributes significantly to successful treatment outcomes. Patients learning to perform self-care at home must learn not only technical details about the PD procedures and the dialysis modality but also new nutritional strategies that are intended to prevent nutritional complications that are all too common in PD patients and contribute to significant morbidity and mortality. PEW, peritonitis, and inadequate dialysis are dreaded complications for PD patients that contribute significantly to poor quality of life, treatment-related morbidity, and illness-related mortality.

The conventional Chinese health education for patients learning PD is initiated in the classroom at the dialysis center and is reinforced through telephone conversations and written materials that are provided to patients regularly (every 1–3 months). This educational strategy has obvious limitations. It is intended to provide life-sustaining knowledge to patients with ESRD, which is accomplished for most patients. However, the education provide consists of a large body of information over a short period, usually 1-2 weeks, and for the most part, it is not reinforced except in cases of treatment-related complications. The standard education does not specifically address the patient's adaptation to chronic illness and the behavioral changes needed to perform PD in the home setting. For many patients, the routine procedure of PD is daunting, and the nutritional requirements are difficult to achieve because the food requirements are so different from the usual Chinese diet. The current Chinese diet is composed of a variety of foods with insufficient high biological value protein, making the traditional culturally derived diet inadequate for the successful management of PD. The current diet with inadequate protein content is heavily influenced by culture, education, and economics, and this is not easy to change. Consequently, PEW is a direct consequence of inadequate DPI and has been associated with adverse clinical outcomes such as chronic inflammation, insufficient dialysis, infection, and accelerated rates of cardiovascular disease.

It has been shown that single and episodic approaches to patient education are not adequate to bring about sustainable behavior change and adherence [13]. Therefore, conventional education is not likely to be enough for the management of young and middle-aged PD patients. In addition to conventional education, our study involves the use of a comprehensive WeChat-based PD education module with a strong emphasis on egg white-based optimal protein intake. WeChat is a widely available social media platform that is flexible concerning the freedom of location and time for communication, and patients could get detailed information through text reading, image sharing, voice communication, and video consultation in WeChat PD groups. Comprehensive PD education is provided through an easy-to-operate mode with greater efficiency and penetration. In addition, the materials are available for repeated review in a socially congruent venue.

The PD nurse sent the pattern of optimal protein intake every 2 weeks and a pattern of comprehensive knowledge about PD every 4 weeks. Similarly, patients sent feedback on their dietary material pictures to the WeChat platform every month under the supervision of medical staff to record the accurate diet of every patient. Nurses command and give prizes to patients who are provided correct feedback on dietary material, point out mistakes of dietary material, and urge the patients who do not send or sent wrong dietary material pictures so that patients follow the physician's dietary recommendation. Furthermore, the problems that patients face in the process of PD are sent to the WeChat group without the limitation of time and location. PD physicians and nurses responded timely. Consequently, both medical staff and patients obtained effective and real information and communicate with each other conveniently. On the other hand, patients who achieve the standard of the recommended diet served as a good model for other patients in the WeChat group. Hence, an increasing number of patients followed the example of the recommended diet, and the intervention is more effectively implemented to attain optimal satisfaction. The results of this study revealed that although the two groups are recommended the same diet, the levels of DPI, EWPI, HBVPI, H/D, and E/H are much higher in IG than in CG. In addition, the dietary adherence rate is better in IG than in CG, while there is no statistical difference in calorie intake in both groups. Therefore, patients in IG are better at incorporating the recommended diet than those in CG because of the use of the comprehensive WeChat-based PD education module.

This dietary intervention takes a particular position on the management of chronic kidney disease (CKD) and its complications. It is a cost-effective treatment and one of the main therapies with evidence of improving serum albumin and prognosis for dialysis patients [14, 15]. The results of our study show better incorporation of the recommended diet by patients in IG in terms of the level of serum albumin attained at 12 months (39.6 ± 3.9 g/L vs. 37.4 ± 3.5 g/L). Moreover, the levels of *Kt*/*V*, Ccr, and RRF are improved in patients in IG than those in CG. The outcome of better dialysis adequacy and residual renal function in the IG can be explained by the improved serum albumin level and nutrition status [16, 17]. The results of the study reveal that patients with DPI < 0.73 g/kg/day have a significantly higher risk than patients with DPI >0.94 g/kg/day in terms of negative nitrogen balance and all-cause and cardiovascular disease mortality. Low-protein intake leads to low protein catabolic rates and is associated with high mortality in patients on dialysis. However, protein is strongly and accurately linked to phosphate, and a protein intake of 1.2 g/kg·d over time is consistently associated with hyperphosphatemia. The risk of death increased by 18% and that of cardiovascular death increased by 10% for every 1 mg/dL increase in serum phosphorus [18, 19]. Hence, restricting dietary phosphorus intake, while increasing DPI is recommended for patients with CKD [20]. Egg white is an unusually rich source of high biological value protein with the lowest phosphate-to-protein ratio and low cholesterol content, and it is a particularly important protein source for patients on dialysis. It is reported that egg white has higher digestibility, biological value, and protein efficiency than other animal and plant proteins. Bioactive peptides such as peptides with antioxidant, antimicrobial, and antihypertensive properties are present in egg-white-related digested products. Treatment of ovalbumin, which is the main ingredient of egg white protein, in water (at 100°C for 5 min) increases digestibility in vitro and simulates human gastrointestinal digestion. Furthermore, because of lifestyle changes, an increase in abdominal fat has become prevalent in impaired glucose tolerance, dyslipidemia, and hypertension, eventually escalating to metabolic syndrome and further to atherosclerotic disease [21, 22]. Moreover, PD patients are at greater risk of these diseases owing to the use of glucose dialysate. Dietary egg white protein, which contains a variety of essential amino acids, is found to reduce body fat mass in rats through an increase in body protein mass. In addition, Taylor's study demonstrated that substituting 8 ounces of pasteurized liquid egg white for meat at one meal per day over six weeks decreased the serum phosphorus level significantly, whereas the serum albumin level tended to increase. For these reasons, an egg white-based diet, which is tender and delicious, can appropriately balance between a high-protein diet to improve PEW and a low-phosphorus diet to avoid hyperphosphatemia. Therefore, intake of 2–4 egg whites by treating in water at 100°C for 5 min every day is strongly recommended. This may facilitate the absorption of egg-white-related digested products, and the increase in EWPI can help avoid excess intake of a high phosphate-to-protein ratio and fat protein. We observed the risk and trend of hyperphosphatemia and hyperkinemia that accompanies an increase in serum albumin-based on dietary egg white protein intake. Lastly, even if the glomerular filtration rate declines to an extremely low level, it still shows a strong inverse relationship with the serum phosphorus level in dialysis [23]. Our data show that patients in IG had better residual renal function than those in CG. The better residual renal function might be one of the reasons why there is no significant difference in serum phosphorus between the groups, whereas the level of DPI is much higher in IG than in CG.

Numerous studies have shown the following findings: RRF can influence nutritional status and serum albumin in patients on dialysis, RRF is an independent factor affecting the hemoglobin level in PD patients, and low serum albumin in patients on dialysis is a predictor of anemia indicating unresponsiveness to conventional treatment for anemia [24]. Another survey reveals that it is difficult to remedy undernourishment in diabetes patients because of the microinflammation, loss of albumin in urine, and accompanying cardiovascular disease. Similarly, the results of the present study reveal a negative relationship between serum albumin and diabetes mellitus and a positive relation with hemoglobin and RRF. Furthermore, our findings reveal the close connection between serum albumin and the ratio of EWPI to HBVPI (*E*/*H*) after adjustment for confounders. This finding facilitates a better understanding of the contribution of egg white-based protein intake to the increase in serum albumin. In our study, in the IG, *E*/*H* in IG arrived at 18.43%, (approximately 19%) at 6 months and further reached 22.34% (exceeding 19%) at 12 months. In the CG, *E*/*H* is 9.8% and 10.19%, respectively, at 6 and 12 months, being significantly lower than those of IG. Consequently, the level of serum albumin in IG is higher than in CG, and the result provides more evidence that egg white-based optimal protein intake could improve the level of serum albumin. However, in this study, the upper limit of the EWPI ratio for improving serum albumin is not confirmed. This may be attributed to the small sample size and the short duration of the study, and further research is needed to explore this possibility.

The young and middle-aged PD patients are rather weak in social and family function, as they had ESRD, which makes patients prone to depression and psychological disorders. The study applies WeChat on smartphones to educate patients on optimal egg white-based protein intake diet in PD, troubleshoot problems, and provide follow-up information. Furthermore, the optimal dietary intervention is integrated with the mental and material motivation that helps patients gain respect and appreciation from others. Motivation may help meet patients' mental needs, foster a positive atmosphere for management, arouse patients' initiative concerning physiology, and increase adherence. Therefore, it can stimulate initiative, improve self-confidence, break psychological barriers, and effectively improve treatment compliance. Additionally, the increased communication with medical staff during the whole intervention process enables young and middle-aged PD patients to gain more health knowledge and support, which enhances their confidence in overcoming the disease. Consequently, the present study shows that the incidence of peritonitis, rehospitalization rate, and scores of KDTA and SF-36 that represent the quality of life in PD patients are much better in the IG than those in the CG.

There are some limitations to the present study. Firstly, it is a single-center, combined prospective and retrospective study with relatively small sample size. Secondly, the patients in the IG are selected randomly, but only half of the patients in the CG can be randomized, necessitating the use of secondary control data to obtain adequate cases for comparison. Furthermore, although all patients are advised to obtain eggs from the supermarket to ensure uniformity, we could not confirm that this happened in all cases. Patients are trained to weigh food, and all food data are self-reported, which could have led to response bias. Nevertheless, this study has several strengths. To the best of our knowledge, the present study is the first to explore the effect of egg white-based optimal protein intake for PD patients. The unique health education platform for young and middle-aged PD patients is designed. Moreover, atleast, this preliminary study points out the associations between serum albumin levels and the ratio of EWPI to HBVPI. Nevertheless, these data can be considered preliminary and additional studies with a larger sample size, and a longer period of observation should be performed to confirm these findings.

## 3. Clinical Treatment Methods and Evaluation Indicators

### 3.1. Patients and Treatment

In total, 115 consecutive new patients with PD between January 2015 and October 2017 are assigned to either the WeChat intervention group (IG) or the classroom control group (CG). We are not successful in the randomization because WeChat is so popular in China that many patients refused to be assigned to the CG. We modify the study to account for the difficulty by adding secondary data of 35 patients as a retrospective CG to the 35 prospectively assigned WeChat CGs from January 2014 to January 2015. Nephrologists and PD nurses followed up with the patients for 12 months after recruitment. Data of clinical and laboratory parameters are collected by a research assistant every 3 months. Informed written consent is obtained from all the participants.  Figure 1 shows the flowchart of the study design.

### 3.2. Interventions and Conventional Education

All patients in both groups received conventional classroom education at the hospital, and any additional patient education is also delivered in the hospital classroom setting. All patients received classroom dietary education emphasizing the need for adequate protein intake. The target DPI of ≥0.8 g/kg, of which at least 50% would be of a high biological value, is the basic recommendation. Chinese PD patients find it challenging to achieve the KDIGO target of 1.2–1.4 g/kg of DPI [25]. In addition to the basic food-derived DPI, all patients received *α*-ketoacidosis supplements at a dose of 5 g/day and are instructed to take 2–4 egg whites per day along with their usual diet. Egg white, which has a very low phosphate-to-protein ratio, is added to help the patients reach the KDIGO dietary recommendations.

Patients in the conventional education (CE) are received conventional education only, which means physicians and nurses performed routine healthy education through telephone calls or oral and sent health text reading materials every 1–3 months.

The conventional education material includes the following aspects: (1) the intake of optimal dietary protein with *α*-ketoacid, and the optimal protein intake is defined as a daily protein intake (DPI) ≥0.8 g/kg·d and at least 50% of the dietary protein should be of a high biological value, through foods such as egg, milk, and lean meat; (2) foods with a low phosphorus-protein ratio (1.2 mg/g) and well-tolerated, 2–4 egg whites, are strongly recommended per day; (3) using of electronic scales to weigh food and record 3-day diary (including 1 working day and 1 weekend); (4) requiring execution of dialysis prescription, operation of dialysate exchange, catheter nursing, self-management, and arrange follow-up time.

### 3.3. WeChat-Based PD Education Module Emphasizing Egg White-Based Optimal Protein Intake (IG)

Patients in the IG have received the same basic conventional education, dietary instructions for a DPI of 0.8 g/kg per day, and 5 g/day of *α*-ketoacid supplement, and they are instructed to supplement their usual diet with 2–4 egg whites per day. The IG, in addition, received a comprehensive PD education module with a strong emphasis on achieving the target intake through 2–4 egg whites daily via WeChat. In addition, the WeChat module provides information on choosing foods with high biological protein content. The comprehensive WeChat platform-based PD education module is carried out by two nephrologists and two PD nurses. The physicians develop the working rules and strategy and regularly summarized and supervised the management of the module. Furthermore, the physicians also design a pattern for this educational intervention module in the form of an easy-to-understand visual image with minimal text forma: (1) the pattern of optimal protein intake is made according to the content of optimal DPI mentioned in conventional education. It also contained visual images of 2–4 egg white intake and the cooking method. This pattern is conveniently sent to the WeChat platform every 2 weeks; (2) the pattern of comprehensive knowledge of PD, such as prevention of peritonitis and self-management, is shared every 4 weeks. The nurses act as the manager to establish the WeChat group and trained the patients who are unfamiliar with the use of WeChat to send or receive messages, voices, images, and videos. In addition, nurses sent the patterns and made group announcements to everyone on WeChat according to the working rules and strategy. At the same time, the patients sent feedback on their dietary intake as pictures through WeChat every month. Then, nurses commended the patients who sent correct feedback on dietary materials and gave prizes. Simultaneously, nurses pointed out mistakes in the dietary pattern so that the patients can correct and send the feedback again and the nurses also urge the patients who do not send the dietary pattern. Furthermore, nurses release follow-up information promptly as planned; (3) patients state the problems that they encounter during PD treatment on the WeChat platform and obtained a response from physicians or nurses within 24 hours in the form of messages, voices, and images.  Figure 2 shows the route of approach for comprehensive PD education on the WeChat platform.

### 3.4. Measurements and Dietary Parameters

Demographic data are collected at baseline, which included age, gender, body mass index (BMI), diabetes, phosphate binders, and *α*-ketoacid. Biochemical indices and dialysis adequacy data are collected at the initial visit, 6 months, and 12 months. Biochemical indices including hemoglobin, serum creatinine, urea nitrogen, serum albumin, and serum lipids are examined by using an automatic chemistry analyzer. In addition, the serum intact parathyroid hormone (iPTH) is tested by isotopic chemiluminescence. The 24-hour urine and dialysate samples are collected to perform the peritoneal equilibration test. Weekly urea clearance (Kt/V), creatinine clearance (Ccr), and normalizing protein catabolic rate (PCR) are calculated using standard methods. Residual renal function (RRF) is estimated using the average renal clearance of urea and creatinine. Data on the incidence of peritonitis, rehospitalization rate, and dietary adherence are recorded during the study. The dietary adherence is calculated using the following formula: the number of patients achieving the recommended dietary protein/total number in the group. Lastly, the feedback rate equaled the actual number of feedback (dietary material picture/the theoretical number), which is recorded only in the IG.

Based on the 3-day diet diary, DPI, egg white protein intake (EWPI), high biological value protein intake (HBVPI), the ratio of HBVPI to DPI (H/D), the ratio of EWPI to HBVPI (E/H), and daily energy intake (DEI) are calculated using the software (Keto Acids Diet Calculator 2.0, China Fresenius). All patients received conventional glucose-based PD solutions (Baxter Healthcare, Guangzhou, China). Total energy intake (TEI) = DEI + calories from dialysate sources [26, 27]. Both DPI and DEI are normalized for standard body weight.

The Kidney Disease Quality of Life-short form (KDQOL-SF version 1.3) questionnaire has been validated for use as a disease-specific measure of the quality of life for dialysis patients and combines the kidney disease-specific instrument (Kidney Disease-Targeted Areas, KDTA) with the generic SF-36 instrument (36-item health survey, SF-36). KDTA has 11 domains with 43 kidney disease-targeted items, including symptoms, effects,and burden of kidney disease, work status, cognitive function, quality of social interaction, sexual function, sleep, social support, dialysis staff encouragement, and patient satisfaction. The SF-36 has 8 domains with 36 generic core items, which are physical function, physical role, pain, general health, emotional wellbeing, social function, energy, and fatigue. The score ranges from zero to 100 with higher scores representing the better-perceived quality of life.

## 4. Comparative Analysis and Data Statistics

In total, 140 patients are enrolled in this study, with 70 in each group. However, 113 patients (59 patients in the IG and 54 in the CG) completed the 12-month follow-up; 11 (15.71%) dropped out from the IG, and 16 (22.86%) dropped out from the CG (Figure 1). No difference in age, education level, sex, BMI, diabetes prevalence, PD duration, dialysate volume, phosphate binders, and quality of life scores are noted between groups. Calcium carbonate is the only phosphate binder used, as shown in Table 1.

### 4.1. Comparison of Dietary Parameters

Both the IG and CG show improvements over time. Thus, the value of dietary protein intake is better in the IG, as shown in Table 2. However, at 6 months, the IG had significantly higher DPI, EWPI, HBVPI, *H*/*D*, and *E*/*H* than the CG, and an interaction effect is also observed (*P* < 0.05). Additionally, this significant difference is maintained at 12 months (*P* < 0.05). No significant difference in DEI and TEI is noted (*P* > 0.05). In Table 2, IG is the intervention group, CG is the control group, DPI is the daily protein intake, EWPI is the egg white protein intake, HBVPI is a high biological value protein intake, H/D is the ratio of HBVPI to DPI, E/H is the ratio of EWPI to HBVPI, DEI is the daily energy intake, and TEI is the total energy intake.

### 4.2. Comparison of Laboratory Parameters

The IG has better value serum albumin levels than the CG at 6 months (*P* = 0.025) and maintains this significant difference at 12 months (*P* = 0.004), and an interaction effect is also observed (*P* = 0.049). The IG also has a significantly higher Ccr, *Kt*/*V*, and PCR and lower triglyceride levels than the CG (*P* < 0.05) at 12 months, but not at 6 months. There is no significant between-group difference in the RRF over time. However, an interaction effect is present (*P* = 0.0112), indicating that the IG had a better time-based value of RRF than the CG. No difference in other parameters is observed between groups, as shown in Table 3. In Table 3, IG is the intervention group, CG is the control group, P is serum phosphorus, iPTH is intact parathyroid hormone, *Kt*/*V* is weekly urea clearance, Ccr is weekly creatinine clearance, and RRF is residual renal function.

### 4.3. Correlation of Serum Albumin Levels with the Ratio of EWPI to HBVPI

Univariate analysis suggested that serum albumin levels are nonlinearly and positively correlated with E/H, H/D, EWPI, HBVPI, and RRF. Moreover, they show a linear and positive correlation between hemoglobin and PCR, and a negative correlation with the presence of diabetes. Threshold effect analysis shows that *E*/*H* (evaluated as a continuous variable) is related to serum albumin levels, and an inflection point *K* is calculated, as shown in Figure 3.

The models are tested using a likelihood ratio test (*P* = 0.005). A segmented regression model is set up with adjustment for confounders such as *H*/*D*, EWPI, HBVPI, RRF, hemoglobin, PCR, and diabetes as follows:

(1) $$\begin{array}{c} Y_{alb}=\beta_{k}\times X_{e/h}+s\left(EWPI\text{ d}f\right)+s\left(HBVPI\text{ d}f\right)+s\left(\frac{H}{D}\text{d}f\right)+s\left(RRF\text{ d}f\right)\\ +\text{hemoglobin}+n\text{PCR}+\text{diabetes}. \end{array}$$

The results are as follows: *E*/*H* ≤ 6.2, *β*_6.2_ = −0.017, 95% CI (−0.488 to 0.454), *P* = 0.944; 6.2 < *E*/*H* < 19, *β*_6.2–19_ = 0.144, 95% CI (−0.03 to 0.317), *P* = 0.106; and *E*/*H* ≥ 19, *β*_19_ = 0.221, 95% CI (0.024–0.419), *P* = 0.029. This suggests that serum albumin levels may increase significantly when *E*/*H* becomes greater than 19%.

### 4.4. Comparison of Peritonitis Rate, Rehospitalization Rate, Dietary Adherence, and Quality of Life

At the end of the study, there is one episode of peritoneal infection for every 0.169 patient-years in the IG, whereas it is 0.333 patient-years in the CG (*P* = 0.047).  Table 4 is the comparison of peritonitis rate, rehospitalization rate, dietary adherence, and quality of life between the intervention and control groups. Meanwhile, the rehospitalization rate is lower, and dietary adherence is higher in the IG than in the CG (*P* < 0.05). Furthermore, the IG received the pattern of optimal protein intake 26 times, and feedback dietary material pictures are to be provided 12 times per patient, resulting in a total number of 708 times. The actual feedback from dietary material pictures is obtained 603 times, and the rate of feedback is 85.15%. Finally, the IG had better KDTA and SF-36 scores than the CG (*P* < 0.05). In Table 4, KDTA is kidney disease-targeted areas, IG is the intervention group, CG is the control group, and OR is the odds ratio.

## 5. Conclusion

This paper uses a comprehensive WeChat platform-based PD education module with a strong emphasis on egg white-based optimal protein intake in addition to conventional education to perform an intensive health education intervention to augment DPI in patients undergoing PD in China. The IG, which receives the WeChat comprehensive education program, not only improves DPI and serum albumin but also robust improvement in clinical outcomes and quality of life, suggesting that the education program engaged the patients and enabled them to participate more in their care to improve dialysis outcomes. Additionally, this study identified an association between serum albumin levels and the ratio of EWPI to HBVPI. A ratio greater than 19% is determined to be the threshold needed to obtain an increase in serum albumin levels. Reinforcing comprehensive PD education using WeChat helps patients, including those with ESRD, improve nutritional parameters, clinical parameters, and quality of life. Education through social media represents a new opportunity for improving prognosis in ESRD patients with PD.

## Figures and Tables

**Figure 1:** Flowchart of the study design.

**Figure 2:** Route of approach for comprehensive PD education on the WeChat platform.

**Figure 3:** Correlation of serum albumin levels with the ratio of egg white protein intake to high biological value protein intake.

**Table 1:** Characteristics of the two groups at enrolment.

Group	Age (years) $\left(\tilde{x}\pm s\right)$	Sex (*N*, (%) men)	Diabetes (%)	BMI (kg/m^2^) $\left(\tilde{x}\pm s\right)$	Education (*N*, (%))		
					Lower than primary school	High school	College degree or above
IG	46.34 ± 13.86	34 (57.63%)	14 (23.73%)	22.95 ± 3.35	6 (10.17%)	37 (62.71%)	16 (27.12%)
CG	48.09 ± 13.40	34 (62.96%)	14 (25.93%)	23.51 ± 3.73	5 (9.26%)	27 (50%)	22 (40.74%)
*t*/*χ*^2^ value	−0.68	0.34	0.07	−0.83	2.38		
*P* value	0.50	0.56	0.79	0.41	0.30		

Group	PD duration (months)	Dialysate volume (*L*/day) $\left(\tilde{x}\pm s\right)$	Ketoacid (g/d) $\left(\tilde{x}\pm s\right)$	Calcium carbonate (%)	KDTA score $\left(\tilde{x}\pm s\right)$	SF-36 score $\left(\tilde{x}\pm s\right)$	
IG	14 (3–27)	7.31 ± 1.39	5.19 ± 3.40	20 (33.89%)	59.74 ± 5.77	52.78 ± 7.46	
CG	9 (5–16)	7.14 ± 1.31	5.78 ± 3.50	17 (31.48%)	58.85 ± 5.49	50.76 ± 7.46	
t/*χ*^2^ value	1.19	0.63	−0.91	0.08	0.83	1.48	
*P* value	0.24	0.53	0.37	0.78	0.41	0.14	

**Table 2:** Dietary parameters from the baseline to the end of the study.

Dietary parameters	Group	0 months	*P* value	6 months	*P* value	12 months	*P* value	Time × group, *P* (coefficient)
DPI (g·kg^−1^·d^−1^)	IG	0.95 ± 0.18	0.59	1.05 ± 0.22	0.02	1.13 ± 0.31	<0.01	0.008 (0.13)
	CG	0.93 ± 0.25		0.94 ± 0.28		0.98 ± 0.30		

EWPI (g·kg^−1^·d^−1^)	IG	0.05 ± 0.04	0.56	0.12 ± 0.05	<0.01	0.16 ± 0.08	<0.01	0.000 (0.09)
	CG	0.04 ± 0.04		0.05 ± 0.05		0.06 ± 0.05		

HBVPI (g·kg^−1^·d^−1^)	IG	0.46 ± 0.13	0.74	0.61 ± 0.21	0.01	0.69 ± 0.23	<0.01	0.001 (0.14)
	CG	0.45 ± 0.19		0.51 ± 0.23		0.53 ± 0.23		

*H*/*D* (%)	IG	47.77 ± 6.45	0.50	56.45 ± 8.85	<0.01	59.73 ± 6.84	<0.01	0.0003 (5.98)
	CG	46.82 ± 8.39		51.95 ± 8.52		52.80 ± 8.51		

*E*/*H* (%)	IG	10.13 ± 6.80	0.57	18.43 + 5.71	<0.01	22.34 ± 7.15	<0.01	0.000 (11.39)
	CG	9.38 ± 7.32		9.82 + 7.62		10.19 ± 7.51		

DEI (kJ·kg^−1^·d^−1^)	IG	110.21 ± 13.74	0.55	111.97 ± 22.35	0.42	117.74 ± 19.76	0.11	0.140 (4.47)
	CG	108.31 ± 19.81		108.52 ± 22.40		111.38 ± 21.75		

TEI (kJ·kg^−1^·d^−1^)	IG	132.36 ± 16.00	0.54	135.90 ± 22.50	0.34	139.09 ± 21.18	0.41	0.422 (2.52)
	CG	130.33 ± 18.93		131.59 ± 25.44		134.54 ± 24.89		

**Table 3:** Change in laboratory parameters from the baseline to the end of the study.

	Group	0 months	*P* value	6 months	*P* value	12 months	*P* value	Time × group, *P* (coefficient)
Albumin (g/L)	IG	36.96 ± 2.87	0.32	38.89 ± 4.00	0.03	39.62 ± 3.85	0.004	0.049 (1.50)
	CG	36.22 ± 4.77		37.02 ± 4.78		37.39 + 3.51		

Hemoglobin (g/L)	IG	102.90 ± 20.21	0.88	101.73 ± 18.24	0.34	104.10 ± 18.81	0.94	0.77 (0.84)
	CG	102.26 ± 22.45		105.59 ± 17.96		103.85 ± 17.10		

P (mmol/L)	IG	1.63 ± 0.49	0.45	1.70 ± 0.50	0.50	1.72 ± 0.38	0.58	0.44 (0.06)
	CG	1.56 ± 0.61		1.62 ± 0.48		1.67 ± 0.48		

iPTH (pg/ml, *M* (P_25_, P_75_))	IG	326.00 (234.80, 481.25)	0.17	350.50 (222.20, 627.10)	0.07	360.20 (217.25, 684.15)	0.12	0.48 (34.63)
	CG	258.60 (138.10, 435.43)		251.60 (133.55, 395.10)		270.10 (100.69, 514.58)		

Total cholesterol (mmol/l)	IG	4.66 ± 1.1	0.82	4.68 ± 1.29	0.60	4.85 ± 1.22	0.85	0.89 (−0.03)
	CG	4.72 ± 1.10		4.81 ± 0.97		4.90 ± 0.93		

Triglyceride (mmol/l)	IG	1.93 ± 1.10	0.76	1.96 ± 1.25	0.40	1.97 + 1.12	0.04	0.07 (−0.50)
	CG	1.85 ± 1.23		2.15 ± 1.21		2.38 ± 1.24		

*Kt*/*V*	IG	2.09 ± 0.49	0.30	1.91 ± 0.45	0.56	1.90 ± 0.32	0.03	0.61 (0.05)
	CG	1.99 ± 0.50		1.86 ± 0.46		1.76 ± 0.39		

Ccr (*L*/week)	IG	67.21 ± 20.08	0.55	59.28 ± 15.79	0.93	59.04 ± 13.17	0.01	0.047 (5.12)
	CG	64.65 ± 25.53		54.61 ± 24.77		52.37 ± 14.09		

RRF (ml/min, *M* (P_25_, P_75_))	IG	2.53 (0.73, 5.36)	0.18	2.29 (0.49, 4.23)	0.79	2.080 (0.00, 4.87)	0.70	0.01 (0.89)
	CG	2.72 (0.56, 6.32)		2.06 (0.34, 4.17)		1.58 (0.34, 3.33)		

nPCR (g·kg^−1^·d^−1^)	IG	0.89 ± 0.20	0.46	0.966 ± 0.185	0.09	1.04 ± 0.19	0.002	0.049 (0.08)
	CG	0.86 ± 0.19		0.881 ± 0.322		0.93 ± 0.18		

**Table 4:** Comparison of peritonitis rate, rehospitalization rate, dietary adherence, and quality of life between the intervention and control groups at the end of the study.

Group	Peritonitis rate (1 episode per patient-year)	Rehospitalization rate (*N* (%))	Dietary adherence (*N* (%))	KDTA score $\left(\bar{x}\pm s\right)$	SF-36 score $\left(\bar{x}\pm s\right)$
IG	0.169	20 (33.9%)	37 (62.7%)	65.44 ± 5.04	59.80 ± 7.46
CG	0.333	28 (51.9%)	15 (27.8%)	61.92 ± 7.56	55.82 ± 5.43
OR/*t* value	0.408	0.476	4.3727	−2.94	−3.25
*P* value	0.047	0.055	0.0003	0.004	0.001

## Data Availability

The simulation experiment data used to support the findings of this study are available from the corresponding author upon request.
